# MicroRNA-200c overexpression inhibits tumorigenicity and metastasis of CD117^+^CD44^+^ ovarian cancer stem cells by regulating epithelial-mesenchymal transition

**DOI:** 10.1186/1757-2215-6-50

**Published:** 2013-07-10

**Authors:** Dengyu Chen, Yunxia Zhang, Jing Wang, Junsong Chen, Cuiping Yang, Kai Cai, Xiaoying Wang, Fangfang Shi, Jun Dou

**Affiliations:** 1 Department of Pathogenic Biology and Immunology of Medical College, Southeast University, Nanjing 210009, China; 2 Department of Microbiology, Bengbu Medical School, Bengbu 233030, China; 3 Department of Gynecology & Obstetrics, Zhongda Hospital, Medical School, Southeast University, Nanjing 210009, China; 4 Department of Oncology, Zhongda Hospital, Southeast University, Nanjing 210009, China

**Keywords:** Epithelial ovarian cancer, Cancer stem cells, MiRNAs-200c, Epithelial- mesenchymal transition, Metastasis

## Abstract

**Background:**

Cancer stem cells (CSCs) are believed to be ‘seed cell’ in cancer recurrence and metastasis. MicroRNAs (miRNAs) can play an important role in the progression of primary tumor towards metastasis by regulating the epithelial-mesenchymal transition (EMT). The goal of this study was to investigate the effect of miRNA-200c overexpression on the EMT, tumorigenicity and metastasis of epithelial ovarian cancer (EOC) CSCs.

**Methods:**

The EOC CD117^+^CD44^+^CSCs were isolated from the human ovarian cancer cell line SKOV3 by using a magnetic-activated cell sorting system, and the lentivirus miR-200c transduced CSCs were then selected for the study. The assays of colony forming, wound healing, cellular migration *in vitro* and tumor progression *in vivo* were performed.

**Results:**

The miR-200c expression was reduced in the CD117^+^CD44^+^CSCs compared with the non-CD117^+^CD44^+^CSCs. However, the stable overexpression of the miR-200c in the CD117^+^CD44^+^CSCs resulted in a significant down-regulation of ZEB-1 and the Vimentin expression, an upregulation of the E-cadherin expression as well as a decrease of colony forming, migratory and invasion *in vitro*. Importantly, the miR-200c overexpression significantly inhibited the CD117^+^CD44^+^CSCs xenograft growth and lung metastasis *in vivo* in nude mice by inhibition of the EMT. In addition, the down-regulation of ZEB-1 showed the same efficacy as the miR-200c overexpression in the CD117^+^CD44^+^CSCs.

**Conclusion:**

These findings from this study suggest that the miR-200c overexpression may be considered a critical approach for the EOC CD117^+^CD44^+^CSCs in clinical trials.

## Background

Ovarian cancer is the leading cause of mortality in gynecologic malignancy. The 5-year survival rate of stage III-IV ovarian cancer patients is about 20% [1,2]. Ovarian cancer is currently treated with a combination of surgery and chemotherapy. Systemic chemotherapy is initially effective in 80% of patients, however, recurrent ovarian cancer’s responds to additional chemotherapy treatments becomes lower after each treatment cycle, as chemoresistance increases until the disease becomes incurable [3]. It is therefore crucial to conduct an in-depth investigation of the biology of ovarian cancer. The major advance of tumor biology in recent years has been the discovery of the cancer stem cells (CSCs), which play pivotal roles in cancer progression and treatment resistance in various neoplastic diseases. CSCs may open up new possibilities of generating novel targets, diminishing resistance to chemoradiation and improving therapeutic efficacy [4].

Tumor metastasis has been considered the main cause of death in patients of various malignant tumors. Evidence from past studies has indicated that the CSC-like cells might be generated by processes that are related to aberrant activation of the epithelial- mesenchymal transition (EMT) that impacts cell differentiation and tumor metastatic potential. Therefore, an anti-EMT strategy would be a novel therapeutic option for treating aggressive cancers [5,6]. There is increasing evidence that the microRNAs (miRNAs) have emerged as potential therapeutic candidates by virtue of their ability to down-regulate multiple targets involved in tumor progression and metastasis, and in tumor therapeutic resistance and relapse. In some studies, miR-200c was found to be down-regulated in ovarian cancer cell lines and in stage III ovarian tumors; the miR-200c down-regulation correlated with poor prognoses. However, restoration of the miR-200c served as a tumor suppressor by directly targeting the zinc-finger E-box binding homeobox 1 (ZEB1) to inhibit EMT and ovarian cancer metastasis [7-10].

The epithelial ovarian cancer (EOC) is genetically and epigenetically distinct from normal ovarian surface epithelial cells and is involved in the EMT during cancer initiation and progression including cancer metastasis and recurrence. ZEB1 is known to be associated with the EOC invasive and metastatic progression; ZEB1 is also known to be expressed in the EOC and be able to directly repress the epithelial marker E-cadherin to induce tumor cell invasive and metastatic progression [11-14]. However, much less information of the EMT is available about the miRNA in the EOC CSCs, and the exact molecular mechanism of modulating the EMT of the EOC CSCs is yet to be elucidated.

Our goal for this study was to assess the epigenetically regulation function of the miR-200c overexpression in the EMT, the tumorigenicity, and the metastasis of the EOC CD117^+^CD44^+^CSCs *in vitro* and *in vivo*. To accomplish this goal, we transduced the lentivirus miR-200c vector into the CD117^+^CD44^+^CSCs that were isolated from the human EOC SKOV3 cell line [15,16]. We found *in vitro* a direct association between the miR-200c overexpression and the capability of the CD117^+^CD44^+^CSC in colony forming, migration and invasion. In particular, we noticed the evident relationship between the miR-200c and the ZEB1 expression. Our results suggested that the miR-200c overexpression, by modulating the EMT, specifically inhibited the ZEB1 expression in the CD117^+^CD44^+^CSCs and reduced cell tumorigenicity and lung metastasis in our nude mouse model.

## Materials and methods

### Cell line

The human EOC SKOV-3 cell line was from an ovarian cancer patient of origin, which was a well-established ovarian cancer model system. The cell line was purchased from the Cellular Institute in Shanghai, China, and was maintained in complete media consisting of RPMI 1640, 2 mM L-glutamine, 100 U/ml penicillin, 100 μg/ml streptomycin, and 10% fetal bovine serum. The complete media were refreshed every 3 days to maintain the adherent cells.

### Isolation of CD44^+^CD117^+^CSCs, transduction of lentivirus miR-200c and production of stable expression colonies

The CD44^+^CD117^+^CSCs were isolated from the SKOV3 cell line by using the magnetic- associated cell sorting (MACS) method as described previously [16,17]. Briefly, the CD44^+^subsets were isolated by using the mouse antihuman CD44 antibody coupled to magnetic microbeads (Miltenyi Biotec., Germany); the resulting cells were then depleted of CD117^−^subsets by using the mouse antihuman CD117 antibody coupled to magnetic microbeads (Miltenyi Biotec., Germany). The resulting CD44^+^CD117^+^cells were labeled ‘EOC CD44^+^CD117^+^CSCs’ [15]. These cells were further identified by using a flow cytometer (FCM, Beckman Coulter, USA) according to the manufacturer’s instructions. The anti-Human/ Mouse CD44 FITC and the anti-Human CD117 PE (eBioscience, USA) antibodies were used for the detection of the cells [18].

To generate the miR-200c expression lentivirus vector, we amplified an insert (full-length human miR-200c) by PCR from SKOV3 DNA. The lentivirus miR-200c was produced from the transient transfection of the HEK293T cells with pHAGE-CMV- miR-200c-IZsGreen, psPAX2, and pMD2.G plasmid DNAs plus Lipofectamine 2000 (Invitrogen, USA) according to the manufacturer's protocol. Forty-eight hours after the co-transfection, the lentivirus-bearing supernatants were collected and passed through a 0.45-mm filter. The CD44^+^CD117^+^CSCs were transduced with the pHAGE-CMV- miR-200c-IzsGreen lentivirus, and were selected by the IzsGreen expression [7,19]. The stable expression colony was generated by limiting the dilution assay [20].

### RNA isolation and quantitative RT-PCR

Total cellular RNA was isolated from a sample by using a Qiagen RNeasy Kit (Qiagen, CA). The sequences of the primers are as follows: the miR-200c-RT primer 5′-CTCAAC TGGTGTGGAGCGCATTCAGTTGAGTCCATCAT-3; the ZEB1 forward, 5′-GCACAAC CAAGGCAGAAGA-3′; reverse, 5′-CATTTGCAGTTGAGGCTGA-3′; the β-actin forward, 5′-GGACTTCGAGCAAGAGATGG-3′; reverse, 5′-AGCACTGTGTTGGCGTACAG-3′; U6: RT Primer, 5′-GTCGTATCCAGTGCAGGGTCCGAGGTATTCGCACTGGATACGA CAAATATGGAAC-3′;forward, 5′-TGCGGGTGCTCGCTTCGGCAGC-3′; URP Universal Reverse Primer, 5′-CCGGCAGGGTCCGAGGT-3′. The E-cadherin forward: CATTGCC ACACATACACTCTCTTCT, reverse: CGGTTACCGTGATCAAAATCTC; the Vimentin forward: GGAACAGCATGTCCAAATCG, reverse: GCACCTGTCTCCGGTACTCA. The qRT-PCR analysis was performed on an ABI step one plus real-time system (Applied Biosystems, USA) [19].

### Short hairpin RNA sequence design and recombinant construction of shRNA1 targeting to ZEB1 gene

A short hairpin RNA sequence of the human ZEB1 was designed according to the ZEB1 DNA sequence (GenBank NO.NM_001128128.2)by the siDESIGN design software of Dharmacon Company. The shRNA sequences were as follows: The ZEB1-siRNA: forward, 5′- GATCCCCAG GAAGAGGAGGAGGATAATTCAAGAGATTATCCTCCTC CTCTTCCTTTTTTGGA AA-3′; reverse, 5′-AGCTTTTCCAAAAAAGGAAGAGGAGG AGGATAATCTCTTGAATTATCCTCCTCCTCTTCCTGGG-3′; the scramble-siRNA: forward, 5′-GATCCCCTTCT CCGAACGTGTCACGTTTCAAGAGAACG TGACACGT TC GGAGAATTTTTGGAAA −3′; reverse, 5′-AGCTTTCCAAAAATTCTCCGAACGTG TCACGTTCTCTTGAAACGTGACACGTTGGAGAAGGG-3′. All the primers were synthesized by Company of Gene and Technology of China in Shanghai. A pSUPER- EGFP1 (enhancement green fluorescent protein 1) vector was used to construct recombinants. The recombinant pSUPER-EGFP1- ZEB1-shRNA (shZEB1) was developed using the method described in a according to previous reports [1,13]. A pSUPER- EGFP1-scrambled shRNA (scramble) was used for negative control. These recombinants were transfected by using the Lipofectamine™ 2000 reagent (Invitrogen, USA) per the manufacturer’s protocol [9].

### Colony forming assay

The colony formation capabilities of the different CD44^+^CD117^+^CSCs were investigated. Colonies larger than 75 μm in diameter or containing more than 50 cells were counted as 1 positive colony according to our previous reports [20,21]. About 500 cells per well were added into a six-well culture plate, with three wells per sample. After12-day incubation, the cells were washed twice with PBS and stained with the Giemsa solution. The plate clone formation efficiency was calculated as (number of colony /number of cells inoculated) × 100%.

### Wound-healing assay

The cells from the above-mentioned colonies were grown to confluence and were wounded by dragging a 1-mL pipette tip across their monolayer. The cells were washed to remove any cellular debris and were then allowed to migrate for 0, 24, and 48 hours, respectively, in a humidified 5% CO2 incubator at 37°C. Images were taken, using a DMI6000 inverted microscope (Leica Microsystems GmbH, Germany), at 0, 24, and 48 hours, respectively, after the wounding procedure [22,23].

### Matrigel invasion assay

The Matrigel invasion assay was done using the BD Biocoat Matrigel Invasion Chamber (pore size: 8 mm, 24-well; BD Biosciences, USA) following the manufacturer's protocol [17,24]. From five randomly selected fields, the cells that had invaded through the membrane to the lower surface were counted under a light microscope.

### Xenograft tumor model

Thirty-six five-to six-week-old female Balb/c athymic *nu*/*nu* mice were ordered from the Animal Center of Yang Zhou University of China and were raised at the Experimental Animal Center, Southeast University. All the animal experiments were performed in compliance with the guidelines of the Animal Research Ethics Board of Southeast University. The 36 mice were randomly divided into six groups of equal size (6) as follows: group 1 for CD44^+^CD117^+^CSCs with lentivirus miR-200c; group 2 for CD44^+^CD117^+^CSCs with lentivirus mock; group 3 for CD44^+^CD117^+^CSCs without lentivirus infection; group 4 for CD44^+^CD117^+^CSCs transfected with the shZEB1; group 5 for CD44^+^CD117^+^CSCs transfected with the scrambled control siRNA; group 6 for CD44^+^CD117^+^CSCs without transfection. Each mouse was subcutaneously (s.c.) injected in the back with 5 × 10^4^ cells for the group it was in. Tumor formations in the mice were monitored every three days. Evaluation was also done of the tumor volume, tumor-free mice, and survival rates, respectively. A mouse was sacrificed when any of its tumors was over 1.4 cm in the largest diameter. The necropsy was performed on each animal for further analysis of the primary tumor along with possible metastases [18,25].

### Western blot analysis

Total cell lysates were prepared and analyzed by using the Western blot method as described before [26,27]. Briefly, 1 × 10^6^ CD44^+^CD117^+^CSCs were collected and lyzed in a protein extraction buffer according to the manufacturer’ s protocol. The PVDF membrane was blocked with 4% dry milk in the Tris-buffered saline with Tween-20 for 1 h at 20°C, and was incubated with the rabbit antibody specific to human ZEB1 (Santa cruz Biotechnology, CA, USA ) or with E-cadherin or with Vimentin (Bioworld Technology, USA) for overnight at 4°C. The membrane was then incubated with the anti-rabbit fluorescence secondary antibody for 1 h at 20°C. Immunoreactive bands were detected by the Odyssey scanning instrument (LICOR Odyssey, USA ).

### Immunohistochemistry

4 μm-thin formalin fixed and paraffin-embedded slides were incubated with the rabbit antibody specific to human E-cadherin overnight at 4°C. The samples were then labeled with HRP-conjugated streptavidin (Invitrogen) and the chromogenic reaction that was developed using Liquid DAB Substrate Pack according to the manufacturer's instructions. E-cadherin-stained cells from random and non-overlapping fields were counted under a magnification of × 200 [28].

### Tissue histopathology

The lung tissues were removed from the mice and fixed in 10% formalin, and then embedded in paraffin. Tissue sections of 4 μm thin were cut and mounted on SuperFrost Plus glass slides, fixed in methanol, and stained in hematoxylin and eosin (HE) [29,30].

### Statistical analysis

Statistical comparisons of the results between groups were performed using the Student’s *t*-test method. *P* < 0.05 was considered significant statistically.

## Results

### Phenotype identification, morphologic characteristics and miR-200c expression in lentivirus transduced CD44^+^CD117^+^CSCs

As was described in the method section, the CD44^+^CD117^+^CSCs were isolated from the SKOV-3 cell line using MACS and were identified for cell phenotype using FCM to study the miR-200c overexpression in CD44^+^CD117^+^CSCs. Figure 1A shows that the CD44 and CD117 double-positive cells accounted for 3.1% of the SKOV-3 cell line, and were labeled ‘CD44^+^CD117^+^CSCs’ as was done before [15]. Next, we detected the miR-200c expression in the CD44^+^CD117^+^CSCs and in the lentivirus miR-200c transduced CD44^+^CD117^+^CSCs after the cells were stably selected using a single clone screening method. Figure 1B indicates that the miR-200c expression analyzed by qRT-PCR was markedly lower in the CD44^+^CD117^+^CSCs than in the non CD44^+^CD117^+^CSCs. The difference was statistically significant (*p* < 0.01). Morphologically, the CD44^+^CD117^+^CSCs transduced with the lentivirus miR-200c appeared to be fusiform-shaped and closely connected clones in the media, whereas the CD44^+^CD117^+^CSCs transduced with the lentivirus mock seemed to have a looser and more dispersed structure (Figure 1C). Figure 1D presents the results of the miR-200c expression analyzed by qRT-PCR. The CD44^+^CD117^+^CSCs transduced with the lentivirus miR-200c (the rightmost bar) exhibited a significantly higher level of miR-200c overexpression than the CD44^+^CD117^+^CSCs transduced with the lentivirus mock (18 ± 5 vs 3 ± 1, *P* < 0.01) or the CD44^+^CD117^+^CSCs (18 ± 5 vs 2 ± 1, *P* < 0.01). Figure 1E presents the E-cadherin expression (brown cells) stained with immunohistochemistry. The results show that more brown cells were found in miR-200c-CD44^+^CD117^+^CSCs of tumor tissue than the control cells.

**Figure 1:** **Identification, selection and detection of the miR-200c expression in the CD44**^**+ **^**CD117**^**+**^**CSCs. A**. The CD117^+^CD44^+^CSCs isolated from the human EOC SKOV3 cell line were identified by FCM; **B**. The miR-200c expression differences between the non CD117^+^CD44^+^CSCs and the CD117^+^CD44^+^CSCs were detected by qRT-PCR; **C**. The top and bottom panels show the morphological structures of the CD44^+^CD117^+^CSCs with the stable miR-200c overexpression under a fluorescence microscope and a light microscope, respectively. The CD44^+^CD117^+^CSCs transduced with lentivirus-mock (left) or lentivirus miR-200c (right) in the stem cell culture medium; **D**. miR-200c expression differences among the CD44^+^CD117^+^CSCs transduced with lentivirus-mock, the lentivirus miR-200c and without lentivirus infection were detected by qRT-PCR. **E**. E-cadherin was detected by IHC assay in tumors of mice injected with the different cells. The labels ‘WT, mock and miR-200c’ denote the CD44^+^CD117^+^ CSCs, the CD44^+^CD117^+^ CSCs transduced with lentivirus-mock, and the lentivirus miR-200c, respectively. These labels are also used in Figures 2, 3, 4 below.

### Effect of miR-200c overexpression on the capability of colony formation and cellular motility of CD44^+^ CD117^+^ CSCs

To characterize the function of miR-200c in the CD44^+^CD117^+^CSCs, we examined the effects of miR-200c overexpression on the CD44^+^CD117^+^CSCs with regard to colony forming, cell migration, cell invasive ability, and cell proliferation ability, respectively. The colony forming capability was analyzed by the plate colony forming assay. The plating colony formation rates were about 60% and 50% for the CD44^+^CD117^+^CSCs and the CD44^+^CD117^+^CSCs transduced with lentivirus mock, respectively; the colony formation rates were less than 20% for the CD44^+^CD117^+^CSCs transduced with the lentivirus miR-200c (Figure 2A, 2D). The cell migration ability was assessed with the wound healing assay; the results are displayed in the pictures in Figure 2B. The overexpression of miR-200c clearly resulted in a significant reduction in cell migration in comparison the control cells (CD44^+^CD117^+^CSCs with lentivirus mock and CD44^+^CD117^+^CSCs without lentivirus infection); the differences were statistically significant (Figure 2E). The cell invasive ability was studied using the transwell invasive assay. The overexpression of miR-200c resulted in fewer CD44^+^CD117^+^CSCs with lentivirus miR-200c (mean ± SD: 70.81% ± 2.16%), in the bottom of the chamber insert, than in the CD44^+^CD117^+^CSCs with lentivirus miR-200c compared with the CD44^+^CD117^+^CSCs with lentivirus mock (125.92% ± 2.14%), or than the CD44^+^CD117^+^CSCs without lentivirus infection (162.26% ± 6.78%) (Figure 2C, 2F). The differences were statistically significant. Figure 2G shows that the proliferation ability of CD44^+^CD117^+^CSCs with lentivirus miR-200c detected by MTT assay was slower than the control cells.

**Figure 2:** **The CD44**^**+**^**CD117**^**+**^**CSCs transduced with lentivirus miR-200c reduced the ability of colony forming, cell migration, invasion and cell proliferation *in vitro*. A**. The plate colony forming assay; **B**. The wound healing assay; **C**. The transwell invasive assay; **D**-**F**. The results of the statistical analysis for the plate colony forming, the wound healing and the transwell invasion, respectively. **G**: The cell proliferation ability of the different cells *in vitro* was detected by MTT assay. *p < 0.05 and ** *p* < 0.01.

### Overexpression of miR-200c reduced ovarian tumor formation and tumor burden

Because the miR-200c overexpression exhibited significant effects on the colony forming and on the migratory and invasion of CD44^+^CD117^+^CSCs *in vitro*, we sought to determine whether the miR-200c overexpression could affect the establishment and progression of ovarian cancer *in vivo* nude mouse model. Figure 3A shows that the growth curves of the tumors in the mice injected with the aforementioned CSCs. The images of the tumors in Figure 3B were taken from the mice injected with the different CSCs when the tumor tissues were dissected on Day 56. Figure 3C indicates the survival time of the tumor-bearing mice. The mice injected with the 5 × 10^4^ CD44^+^CD117^+^CSCs with lentivirus miR-200c showed much higher tumor free rates than the mice injected with the 5 × 10^4^ CD44^+^CD117^+^CSCs with lentivirus mock or 5 × 10^4^ CD44^+^CD117^+^CSCs without lentivirus infection on different days after the injection. The differences were statistically significant (*p* < 0.01 in both comparisons). The results suggested that the stable miR-200c overexpression in established tumors delayed tumor progression.

**Figure 3:** **The miR-200c overexpression decreased tumor progression of CD44**^**+ **^**CD117**^**+ **^**CSCs in xenograft mice. A**. 5 × 10^4^ CD44^+^CD117^+^CSCs transduced with lentivirus miR-200c or lentivirus-mock or without infection were subcutaneously injected in the nude mice ( n = 6/group). The figure shows the tumor growth dynamic state in the mice injected with the different CSCs (line, mean ± SE). **B**. Images of the tumor tissues dissected from the mice on day 56 after injection. **C**. Tumor-free mice on day 56 after injection(line, mean ± SE). *p < 0.01 and ** *p* < 0.01.

### miR-200c inhibited ZEB1,Vimentin and enhanced E-Cadherin expression levels in tumor as well as decreased tumor lung metastasis in nude mouse model

It is known that the feedback loop model links ZEB1 to miR-200c in melanoma and breast cancer cells, and that ZEB1 and miR-200c repress each other in the loop that impacts the change in EMT-MET[10,23]. Therefore, we wanted to find out whether the miR-200c overexpression would also impact the ZEB1 expression in the tumors of the nude mice that were injected with the CD44^+^CD117^+^CSCs with lentivirus miR-200c. The results revealed that the miR-200c overexpression in the tumors led to a marked reduction of ZEB1 mRNA (Figure 4A), Vimentin mRNA (Figure 4B) and the protein expressions (Figure 4D) compared with the CD44^+^CD117^+^CSCs with lentivirus mock and with the CD44^+^CD117^+^CSCs without lentivirus infection. Figures of 4E to 4G present the quantities of the molecular expression from the gradation scanning analysis. The miR-200c overexpression in the tumors significantly increased the E-cadherin expression (Figure 4C, 4F). Because the stable miR-200c overexpression in the established tumors delayed tumor progression and extended the survival of the tumor-bearing mice, we wanted to find out if the miR-200c overexpression would inhibit tumor metastasis. Figure 4H shows that the tumor lung metastasis was significantly reduced in the mice injected with the CD44^+^CD117^+^CSCs with lentivirus miR-200c in comparison with the mice of the two control groups (Figure 4I).

**Figure 4:** **Impacts of the overexpression of miR-200c on ZEB1, E-Cadherin, and the Vimentin expressions in tumors, and tumor cell metastasis in mouse lungs. A**-**C**. The qRT-PCR analysis results of the mRNA expression of ZEB1, Vimentin and E-Cadherin in the tumor tissues of EOC-bearing nude mice after injection with CD44^+^CD117^+^CSCs. **D**. The protein expression of ZEB1, E-Cadherin and Vimentin from the Western blotting analysis. **E**-**G**. The protein expression results from the gradation scanning analysis. **H**. The tumor metastasis in mouse lungs (stained in hematoxylin and eosin). **I**. The statistically significant differences are indicated by asterisk for **p < 0.01.

### Effects of down-regulation of ZEB1 on colony formation, migration, invasion of CD44^+^CD117^+^CSCs in vitro, tumorigenicity, and tumor metastasis *in vivo*

Figure 5A displays the results from our experiment that investigated the effects of the down-regulated ZEB1 expression on the CD44^+^CD117^+^CSCs. The shZEB1 CD44^+^CD117^+^CSCs significantly decreased the colony forming rates compared with the CD44^+^CD117^+^CSCs and the scrambled CD44^+^CD117^+^CSCs, respectively; Figure 5D indicates that the differences were statistically significant (*P* < 0.01). Further, we evaluated the cell migration ability in the shZEB1 CD44^+^CD117^+^CSCs. Figure 5B gives the representative images of the cell migration in the flat plate. The shZEB1 CD44^+^CD117^+^CSCs obviously slowed the cell migration due to the scratchy ‘wounds’ at the cell edges. The results from the quantitative analysis at 48h showed a statistically significant reduction in the wound closures in the shZEB1 CD44^+^CD117^+^CSCs compared with the CD44^+^CD117^+^CSCs and the scrambled CD44^+^CD117^+^CSCs, respectively. Figure 5C illustrates the cell invasive ability of the shZEB1 CD44^+^CD117^+^CSCs as was measured by the transwell invasive assay; the differences between the shZEB1 CD44^+^CD117^+^CSCs group and the other two groups were both statistically significant (*P* < 0.05 and *P* < 0.01 as shown in Figure 5F).

**Figure 5:** **Down-regulation of ZEB1 inhibited the colony forming, cell migration and invasion *in vitro*. A**-**C**. The representative images from the results of the plate clone forming assay, the wound healing assay, and the transwell invasive assay, respectively; **D**-**F** give the between-group statistical differences in the plate colony forming ratio, in the healing degree, and in the invasive cells, respectively. The labels ‘WT, scramble and shZEB1’ denote the CD44^+^CD117^+^CSCs, the CD44^+^CD117^+^CSCs stably transfected with scramble shRNA, and the CD44^+^CD117^+^CSCs stably transfected with shZEB1, respectively. *p < 0.05 and **p < 0.01. These labels are also used in Figure 6 below.

In light of the observed effects of the decreased ZEB1 expression on colony forming, cell migration and invasion in the shZEB1 CD44^+^CD117^+^CSCs *in vitro*, we further validated whether the effects would impact the tumorigenicity and metastatic potential of the shZEB1 CD44^+^CD117^+^CSCs *in vivo*. Figure 6A shows that all the 6 mice in this group developed tumors in 20 days after the injection of the 5 × 10^4^ CD44^+^CD117^+^CSCs; 5 of the 6 mice in the group receiving the 1 × 10^6^ scrambled cells developed tumors in 26 days after the injection. In contrast, only 3 of the 6 mice injected with the 5 × 10^4^ shZEB1 CD44^+^ CD117^+^CSCs developed tumor on Day 22, Day 26 and Day 28, respectively; the other 3 mice did not grow tumors throughout the 56-day observation period (Figure 6B). Figure 6C displays the photos of the tumor sizes and quantity in the mice when the resultant xenograft tumors were harvested.

**Figure 6:** **Down-regulation of ZEB1 reduced tumor growth and metastasis *in vivo *xenograft mouse. A**-**B**. The tumor dynamic growth curves and tumor bearing mice’ survival. **C**. The photos of the tumor tissues dissected from the mice on day 56 after injection. **D**. The protein expression results from the Western blotting analysis. **E**-**G**. The protein expression results from gradation scanning analysis. **H**. The HE staining results from the tumor tissue sections at 400× magnification; The tumor cell metastases were visible in the samples of the CD44^+^CD117^+^WT(+++) and the CD44^+^CD117^+^ scramble (+++); a few tumor cells were seen in the lungs of the nude mice injected with the CD44^+^CD117^+^shZEB1 (+). I.The statistical analysis results of the metastatic tumor cells in the lungs of the mice injected with the different CSCs. *p < 0.05 and **p < 0.01.

To characterize the function of the downregulation of ZEB1, we examined the expression of ZEB1, E-cadherin and Vimentin, respectively, in the tumor tissues of the EOC-bearing nude mice. The Western blot results indicated that the expression of ZEB1 and Vimentin was much lower, and the E-Cadherin expression was much higher in the mice injected with the shZEB1 CD44^+^CD117^+^CSCs than in the mice injected with the CD44^+^CD117^+^CSCs or with the scrambled CD44^+^CD117^+^CSCs (Figure 6D). Figures 6E to 5G show the quantities of the molecular expression from the gradation scanning analysis.

To assess the effect of the down-regulation of ZEB1 on tumor metastasis, we performed H&E staining of lung tissue sections. Compared with the mice of the two control groups, a few tumor metastasis were found in the lungs of the nude mice injected with the shZEB1 CD44^+^CD117^+^CSCs (Figure 6H and 6I). It is thus evident from the results that the EMT-phenotype tumor cell growth and metastasis were significantly inhibited in the mice injected with the shZEB1 CD44^+^CD117^+^CSCs compared with the mice injected with the CD44^+^CD117^+^CSCs or the scrambled CD44^+^CD117^+^CSCs.

## Discussion

EOC CSCs that undergo the EMT have demonstrated that the tumor cells are in general less differentiable, more invasive, more chemoresistant, and result in poor clinical outcomes [7]. Numerous studies of EOC have focused on modulating the miR-200 family (including miR-200a, miR-200b, miR-200c, and miR-141) [31-34]. However, it is unknown whether the EOC CSCs, the “seed cells” in EOC, are closely associated with the miR-200 family expression.

The findings from our study demonstrated that the population of the rare CD44^+^CD117^+^CSCs (3.1%) existed in the human EOC SKOV3 cell line, and that the CD44^+^ CD117^+^CSCs showed lower expression of miR-200c than the non CD44^+^CD117^+^CSCs. With the stable miR-200c overexpression in the CD44^+^CD117^+^CSCs, the cells markedly decreased the colony forming capability. It is known that the tumor cell cloning efficiency is correlated positively with the cellular proliferation and self-renewal ability that may be associated with the cell tumorigenesis [23,24]. The results from our colony forming assay indicated that the small subset of the CD44^+^CD117^+^CSCs had a strong colony forming capability, which signified that the CD44^+^CD117^+^CSCs might have powerful tumorigenesis in the mouse model. In our tumorigenesis analysis, we found that all 6 nude mice injected with the 5 × 10^4^ CD44^+^CD117^+^CSCs developed tumors in 21 days after the injection. In comparison, for the group that was injected with the 5 × 10^4^ CD44^+^ CD117^+^CSCs with the miR-200c overexpression, only 3 out of the 6 mice with equal injection of 5 × 10^4^ cells developed tumors after 56 days into the observation; the tumor sizes of these 3 mice were also smaller than those of the control group mice. These results suggested that the miR-200c overexpression not only effectively decreased the colony forming capability but also obviously reduced the tumorigenicity and the tumor burden in our establishment mouse model.

In EOC, metastases account for the majority of deaths from gynecologic malignancies [35,36], therefore, we next explored the relationship between the miR-200c overexpression and tumor metastases. The cell migration and invasion *in vitro* results indicated that the stable miR-200c overexpression in the CD44^+^CD117^+^CSCs reduced cell migration and invasion. It is well known that the cell migration and invasion *in vitro* are definitely associated with of cell metastases *in vivo*; this was confirmed by the lung metastasis in the mice in our study. The lung tumor metastasis in the mice injected with the CD44^+^CD117^+^CSCs with lentivirus miR-200c was markedly decreased. To study the efficacy of decreased tumor metastasis in the lungs of the mice in the study, we wanted to understand what molecular mechanism of reduced the tumor metastasis; we investigated this by detecting the characteristic biomarkers of E-cadherin (epithelial cells),Vimentin (mesenchymal cells), and ZEB1 (in association with EMT) in tumor tissues [9,37]. We noticed that the enforced overexpression of miR200c in the CD44^+^CD117^+^CSCs significantly reduced the expressions of both ZEB1 and Vimentin, but increased the expression of E-cadherin in the RNA and the protein levels in tumor samples. Apparently, the miR-200c overexpression decreased the ZEB1 expression, which directly inhibited the EMT of the CD44^+^CD117^+^CSCs, and reduced the CSC metastasis potential. Our findings were in agreement with a recent report that the overexpression of miR-429, a member of the miR-200 family of microRNAs, in the mesenchymal-like ovarian cancer cells resulted in the mesenchymal–epithelial transition [33].

To assess the relationship between ZEB1 and miR-200c in the CD44^+^CD117^+^CSCs, we asked whether the down-regulation of ZEB1 would have similar effects as the miR-200c overexpression. We found that the down-regulation of the ZEB1 expression in the CD44^+^CD117^+^CSCs indeed had the similar effects as the miR-200c overexpression in the CD44^+^CD117^+^CSCs; this was reflected in the significant suppression of the tumorigenesis and tumor metastasis in the mice injected with the shZEB1 CD44^+^CD117^+^CSCs in comparison with the mice injected with the CD44^+^CD117^+^CSCs or with the CD44^+^CD117^+^CSCs with lentivirus mock. It is therefore reasonable to conclude that ZEB1 was essential for tumorigenesis and metastasis in xenografts transplantation experiments, and that the down-regulation of ZEB1 may not only be a useful biomarker of the EMT in the EOC CSCs, but also serve as a potential therapeutic target to inhibit EOC metastasis [33,37].

In summary, the findings from our experiments demonstrate that the overexpression of miR-200c significantly reduced the CD117^+^CD44^+^CSCs xenograft growth and lung metastasis *in vivo*, partially through the reversal of the EMT phenotype. The down- regulation of the ZEB-1 expression in the CD117^+^CD44^+^CSCs induced the similar effects as the miR-200c overexpression. These findings may enable us to design a feasible strategy for the modulation of EMT in the CD44^+^CD117^+^CSCs for clinical EOC treatment.

## Competing interests

The authors declare that they have no competing interests.

## Authors’ contributions

DC, JW and YZ carried out the experiments described in the manuscripts, developed the technique described in the manuscript, and participated in the writing of the manuscript. JC, CY, KC, XW, and FS participated in most of the experiments. JD contributed to the design of the experiments and to the writing of the manuscript. All authors have read and approved the final manuscript.
